This article has been retracted.

# The Influence of Disney Musical Practice Course on the Mental Health of Chinese Left-Behind Children from the Perspective of Art Communication

**DOI:** 10.1155/2022/5738531

**Published:** 2022-06-24

**Authors:** Wei Cao

**Affiliations:** ^1^School of Art, Southeast University, Nanjing, Jiangsu 211189, China; ^2^School of Theater, Film and Television, University of California, Los Angeles (UCLA), Los Angeles, CA 90095, USA

## Abstract

**Background:**

In recent years, with a large number of rural people going out to work, the mental problems of left-behind children have been widely concerned by people from all walks of life.

**Objective:**

The purpose is to improve the teaching quality of music education of left-behind children and solve their unique mental problems.

**Methods:**

Based on the questionnaire survey, the mental state of left-behind children is studied, and the mental problems of left-behind children are intervened based on musical practice classes. First, the left-behind children's mental status is studied. Second, through the questionnaire, the left-behind children's music classroom status is studied and analyzed. Then, the musical classroom intervention experiment is designed to prevent and adjust the left-behind children's mental problems.

**Results:**

The results show that more than 90% of left-behind children spend less than one month with their parents every year. Most of the left-behind children are supervised by their grandparents, and 68% of them have been accompanied by their grandparents for more than nine months. Due to the lack of parents' company, most of the left-behind children are lack of self-confidence and timid and tend to care about others' opinions. Musical practice classes have a good effect on the regulation and prevention of left-behind children's mental problems.

**Conclusions:**

This study uses a questionnaire survey method to explore the new form of left-behind children's music classroom, preventing and regulating left-behind children's mental problems, which provides a reference for the research in related fields.

## 1. Introduction

With the accelerated pace of urban modernization, more and more rural residents go to the city for a living, leading to the phenomenon that the number of left-behind primary school students is increasing. This is rapidly evolving into a social problem, causing a series of mental problems such as education problems and emotional problems [1, 2]. Because primary school students are young and have a strong dependence on their parents in emotion and life, the rapid changes in the family environment lead to more and more mental problems of left-behind primary school students. The lack of emotional care and cultivation during the growth process contributes to some differences in understanding and values from others, as well as psychological abnormalities, which is easy to make them commit crimes [3]. Due to the lack of care from their parents, left-behind children suffer from different degrees of physical and mental problems. In this case, schools should provide appropriate care and education to provide a healthy environment for left-behind children. They adopt music intervention and other disciplines and choose the best music content and intervention path to provide a strong guarantee for the development of children's physical and mental health [4].

Some researchers believe that the mental problem of primary school students is the interruption of emotional maintenance [5]. Long-term separation from their parents makes them lack the necessary emotional attachment with their parents, which easily leads to emotional separation from their parents [6]. The surrogate guardian is also difficult to detect their emotional changes so that left-behind children miss the most basic mental communication opportunities. This long-term emotional accumulation is easy to make left-behind children show the extreme personality of inferiority, pessimism, seclusion, or depression, and make their social problems [7, 8]. The influence of parents' work on the left-behind children is complex. With the growth of age, left-behind students gradually realize the importance of family and parental care, and their satisfaction with life gradually decreases. The lack of parent-child education makes children keener on parental comfort and attention [9, 10]. This feeling is easy to produce mental pressure, which leads to depression, discomfort, or lack of opinion. These negative emotions are not conducive to the development of physical and mental health and easy to form mental problems, leading to the development of unhealthy personality. Toropova (2020) [11] pointed out that with the rapid development of information technology, various forms of cartoons appeared rapidly, which had begun to affect the learning and life of the new generation of children. Cartoons have the characteristics of real and vivid characters, rich and colorful content, bright colors, and strong rhythm. They can make difficult and abstract content simple and easy to understand, helping to maintain children's mental health. Hove et al. (2022) [12] pointed out that cartoons can also mobilize students' initiative in learning. When primary school students are learning, they will inevitably have feelings of fear and boredom, and teaching should make primary school students actively learn and explore. More importantly, primary school students acquire knowledge in a happy mood, and these characteristics of cartoons meet the needs of students' development. Madden and Jabusch (2021) [13] pointed out that positive psychology is a discipline concerned with human well-being and health. As a supplement to psychology, positive psychology mainly focuses on people's positive conditions, taps people's positive potential, and returns to people's rationality. Psychology traditionally focuses on the current state of negative and pathological psychology, while positive psychology embodies the spirit of the times. Through the research analysis on left-behind children and their psychological status, the research on the psychological problems of left-behind children in rural areas is a branch of children's psychological problems. Children's psychological problems are often associated with personality, behavior, moral development, academics, family, and school education. Psychological problems are not isolated problems but systemic social problems. Most studies show that left-behind children have psychological problems, and their mental health status is different from that of non-left-behind children. For the differences, more emphasis is placed on the lack of parent-child relationship and the incomplete family education function. The countermeasure research basically focuses on family education and emotional care reinforcement, school education quality, and social support.

This study takes lower-grade primary school students as the research object. Through the questionnaire survey method, the educational function contained in the Disney musical curriculum is analyzed and summarized. The innovation and contribution are that with the technical support of the modern Internet, the Disney musical course is applied to the research on the impact of left-behind children's mental health. This study provides a certain reference value for applying for Disney musical courses in the study of left-behind children's mental health.

## 2. Theory and Method of Teachers' Ethics

### 2.1. A Study on the Psychological Status of Left-behind Children

1. From the perspective of mental health, many left-behind children are faced with huge mental pressure and growth risks, such as emotional vulnerability, self-abandonment, anxiety and autism, lack of self-confidence, pessimism, and negative and other mental problems due to the lack of care from parents, as well as the influence of economic conditions, public security environment, social environment, and other factors. Some even appear mental abnormalities. Parents play a very important role in the growth of children. When parents go out to work, left-behind children grow up in the environment of long-term lack of parental care, which will make them feel lost and lonely, making them becoming self-abased and autistic because they lack the communication, help, and advice they need in their daily lives. And then they have feelings of helplessness and low self-esteem. This is very harmful to the healthy growth of left-behind children
2. In terms of moral quality, without supervision and self-control, the left-behind children are easy to be affected by the external environment, so that there appear various problems in students' moral quality. This causes them to lack moral senses, honesty to others, being grateful, relying heavily on family and friends, indifference to neighbors and society, and even lack of social responsibility
3. In their daily lives, the left-behind children do not have a competent guardian. Some left-behind students are willful, selfish, and have bad habits. In addition, most of the children have personality disorders, such as indifference, introversion, loneliness, and inferiority. Their behavior problems are mainly that they follow their inclination, disobeying discipline, violating school discipline, and even participating in some illegal and criminal activities. They also have difficulty in communicating with others and cannot actively participate in collective activities [14, 15].
4. In terms of their characters, the left-behind children's personality traits are cold and lonely because of their lack of parental education, emotional instability, and poor self-control. They often feel inferiority, apathy, depression, anxiety, and irritability

The main reason for the negative emotional problems of left-behind children is that their parents' long-term absence makes their physical and mental needs cannot be met and their emotional problems are mainly manifested in four aspects [16, 17]: (1) loneliness; (2) sensitivity and inferiority; (3) strong anxiety; and (4) grievance and sadness.

In addition to the above, the unhealthy emotions of left-behind children are also reflected in the following behaviors, including playing a trick on others, disobeying disciplines, reluctant to participate in social activities, and having difficulties in communicating with others. The behaviors are related to the age of left-behind children; the younger the children are, the more such behaviors they have. Positive emotions promote people's cognitive activities, making people feel comfortable, cheerful, optimistic, and confident, while negative emotions make people feel depressed, thereby influencing their mental health [18]. Lack of long-term emotional experience brings strong negative emotional experience to left-behind children, which leads to the lack of social responsibility of left-behind children [19].

### 2.2. The Theoretical Basis of the Positive Influence of Music Education on Left-Behind Pupils

The mental process between music education and music practice course is a mental process in the development stage of personality traits and basic music knowledge and skills of the educated, which is closely related to human development [20]. The establishment of education systems needs to be based on the change of people's mental activities, so the curriculum design and practice of modern education should not be separated from psychology. It is necessary to better understand the characteristics of students' psychological activities and master the process and laws of students' psychological development to create an atmosphere conducive to the healthy and all-around development of students. The goal and content of music education should match the various stages of students' physical and mental development [21]. The cultural psychology of music education has a strong appeal in terms of academic foundation, values, and changes in postmodern philosophy [22, 23]. Many international music education studies offer different methods of music teaching. The concept of music education comes from musicology, pedagogy and psychology, social science and anthropology, and other related disciplines. The emergence of these humanities provides a variety of theoretical and practical data to study the deep-seated problems of music education.

### 2.3. Research Methods

With the rapid development of science and technology, people's life needs have been satisfied. People began to pay attention to their own state of mind. Zheng et al. (2020) pointed out in the study that overprotection makes children's creativity decline, which is an unconscious injury. However, lacking care may also hurt children [24]. This study is to explore and study the mental problems of left-behind children caused by the lack of their parents' company.

Through the literature research method, the important role and significance of music practice courses for left-behind children in primary school are analyzed. Relevant music education methods and other theoretical knowledge related to educational psychology research literature are reviewed to understand the current situation of music education for left-behind children in rural areas, improving the people's professional theoretical knowledge reserve. And the problems and deficiencies in music education for left-behind children are scientifically analyzed [25–27]. The effective methods to improve the learning status of left-behind children provide a valuable reference for the feasibility study on the left-behind children, finding a scientific solution to the problem.

### 2.4. The Role of Musical Practice in Music Education

Music is a natural form of expression and an organic part of human spiritual life. In the daily music education classroom, there are a lot of skills and subjects that need to be taught. Music education and children's education should be combined with learning and experience, focusing on children's participation in music experience and practice. Music education does not need to understand basic music knowledge and skills as a single educational content but needs to reintegrate with other relevant educational media and social resources, adapting to the development of the times [28, 29].

Music can transfer the beauty of art. Playing music has two basic characteristics: notes cannot directly reflect the visual image, and language cannot directly express the concept. Appreciate music from the angle of music aesthetics, which makes the grammar here clearer and clearer. Music is also a living art reflecting social reality to realize one's values. Music works of different times can reflect the author's social development and cultural and historical context through the author's feelings and life experience [30, 31]. Music education must integrate music practice into classroom teaching to cultivate students and discover the beauty of music in the process of listening. The types of music practice can be summarized as the process of sublimating music learning, such as singing, playing instrumental music, reciting game score, and impromptu performance. This training mode can avoid boredom. Mechanical songs can cultivate children's long-term interest in rich and colorful music forms. Music art practice course is an extension of music course. In the process of performance, learners show the audience the music and artworks they have learned, understood, or created in the music practice. These connections not only enable learners to better understand the basic principles of music but also better promote their independent learning initiative. A rich and colorful music practice course is an important way to maximize the value of university music education and an important part of moral and art education. In primary school music teaching, students can listen to music by creating their melody in a comfortable environment through music practice. It can fully extend the core values of general music class and cultivate the students' enthusiasm and initiative [32, 33].

In addition to the development of students' innovative psychology, musical practice courses can also promote cooperation, communication, and expression of basic skills between teachers and students. Music education can help enrich emotion, shape temperament, and develop students' intelligence. Through the communication and education in music practice, most left-behind children love and accept music very easily, which will bring different psychological reactions for some children and reduce their depression and eliminate anxiety. Some children can open their hearts and create music that suits their emotions. The comprehensive training of students' music practice ability can develop their creative thinking, enrich their imagination, and stimulate their creativity. Music practice teaching is an important part of music education in primary and secondary schools, and its organizational form is flexible. The practice content is more diversified than the general music class, which can better integrate the knowledge between different disciplines, such as the ability to express themselves and describe pictures.

### 2.5. Main Characteristics of Disney Musicals

Musicals are also called stage plays. It is a form of stage performance with performance as the carrier. Through this form of performance, the audience will be more easily integrated into the situation and emotionally resonate with the performer. The stage play also plays a very important role in improving the appreciation level of the viewers. A common problem in primary school teaching is that students have difficulty concentrating. Elementary school students are relatively young and have not yet formed mature thoughts, and their behaviors are greatly affected by external influences. They are easily distracted by other things in the classroom learning process, and it is difficult to maintain a high degree of attention in the classroom. On the other hand, students do not recognize the importance of learning, have low interest in learning, and have low classroom participation. This will have a very negative impact on improving students' appreciation and aesthetic level and hinder the realization of primary school music teaching goals. In recent years, Disney musicals have swept the world and have had a profound impact on children's musicals worldwide. The main characteristics of Disney musicals can be divided into three points.

#### 2.5.1. Playful

An important feature of Disney musicals is that they are playful. It is not only loved by “small audiences,” but also can stimulate the “innocence” in the hearts of adults. Disney musicals strongly highlight the characteristics of childishness and integrate them into the perfect, making the audience feel the beauty of childhood when watching the performance.

#### 2.5.2. Teach through Lively Activities

This education method originated from the Disney musical in the USA, adhering to the American education model. American spirit and patriotic education are integrated into the musical. The main audience of Disney musicals are children and families, which should not be too “childlike,” but reflect the essence of education. While bringing joy to children and parents, musicals also achieve the role of “assimilation” of values and outlook on life. The American spirit it promotes mainly includes freedom and equality, hard work, and discerning right from wrong. These American spirits are perfectly expressed in the Disney musical and recognized throughout the country and the nation. Today, Disney is deeply affecting people around the world.

#### 2.5.3. The Production Lineup Is Huge and Luxurious

The artistry of Disney musicals is worthy of admiration in the world. Still, in the process of advocating art, its inherent commerciality and popularity cannot be denied, especially in a market economy environment. In order to meet the needs of a wider audience, Disney musicals often have a strong lineup and magnificent stage effects, giving the audience a strong visual impact. After hundreds of years of accumulation and precipitation, most of the musicals launched by Disney are grand and gigantic productions. Among them, advanced technological equipment will create a beautiful stage landscape.

### 2.6. Questionnaire and Research Design

A school in China is sent out a questionnaire. In order to understand the physical and mental conditions, students of left-behind children in an experimental school in the urban-rural fringe of a province in China are surveyed on the actual situation. Students in the lower grades are selected as the most representative research subjects, 293 questionnaires are distributed to the lower grades, and 270 valid questionnaires are recovered. The effective rate of the questionnaire is 92.1%. Then, the survey data is collected and organized. Office software is used to perform scientific analysis and calculation of the collected data. The detailed information lays a solid foundation for the following research work. This survey is conducted with the consent of the participants and guardians. The research data and results are only used for this study and are not used for other purposes.

SPSS 26.0 is used for the reliability analysis of the questionnaire, and Cronbach's alpha is 0.804. It is larger than 0.7 and has good reliability. The reliability statistics results are shown in Table 1:

SPSS 26.0 is used to perform Kaiser-Meyer-Olkin (KMO) and Barlett tests on the questionnaires. Thus, the questionnaire is subjected to factor analysis, and the validity of the questionnaire is obtained. The KMO is 0.657, which is greater than 0.6. Each question in the questionnaire is suitable for factor analysis and has good construct validity. The tests of KMO and Bartlett are shown in Table 2.

This questionnaire has good reliability and validity, and the student survey data is reliable.

## 3. Questionnaire Results and Analysis

### 3.1. Survey Results of the Basic Information of Left-behind Children

The basic information of left-behind children is shown in Table 3.

According to the gender and age of the investigated organic children shown in Table 1, there are 58 left-behind children in grades 1 and 2. Among the 58 left-behind children, there are 36 boys, accounting for 62.09% of the total number of left-behind children. There are 22 girls, accounting for 37.1. Among them, 82.7% of the students are under 7 years old, and most of the oldest students are about 8 years old. According to the survey on their guardians, 84.4% of children are under the guardianship of grandparents, 8.6% of them are under the guardianship of grandparents-in-law, and 7.0% are under their relatives.

The company of left-behind children throughout the year is shown in Figure 1.

Figure 1 shows that more than 90% of left-behind children spend less than one month with their parents each year. Most of the left-behind children are supervised by their grandparents, 68% of them are accompanied by their grandparents for more than nine months, and 17% for more than half a year. It is found that the left-behind children are extremely short of their parents' companionship.

### 3.2. Investigation on the Mental Health of Left-behind Children

The mental health states of left-behind children are shown in Figure 2.

Figure 2 shows that nearly 90% of the left-behind children often miss their parents. 75% of left-behind children often feel lonely and insecure. They think other children are better than themselves. 60%-70% of left-behind children think that they sometimes lie and have a bad temper. More than 50% of left-behind children sometimes feel afraid and helpless. On this basis, it is concluded that most left-behind children lack self-confidence, are timid, and easy to care about others' opinions.

### 3.3. A Survey of Left-Behind Children's Understanding of Music Classes

The attitudes of left-behind children towards music classes are shown in Figure 3.

Figure 3 shows that more than 90% of the left-behind children like music very much. 87% of the left-behind children argue that they like music lessons very much. More than 90% of the children believe that they like the music teacher very much, while less than 50% of the left-behind children like to sing, perform, and answer questions frequently. This shows that left-behind children like music and singing, and think music can make them relax and be happy, but many of them are shy to perform and express themselves in public because of their introverted characters and timidity.

The reasons for left-behind children's liking of music lessons are shown in Figure 4.

Figure 4 shows that most children like music class because they like the music itself. Many students like music classes because it is easy and interesting and they like music teachers. Less than 5% of students do not like music classes. In terms of the content of music classes, most students think that music classes can play a role in cultivating moral character and help them understand the local customs of a place. With regard to the teaching method of music classes, most students like singing and practice.

The music knowledge of left-behind children is shown in Figure 5.

Figure 5 shows that only about 30% of the left-behind children can understand the knowledge of the music theory in the music textbook, and most of the other students only understand part of it. However, with the intervention of music practice classroom for four months, the number of children who cannot understand the knowledge of the music theory is gradually decreasing, and the number of students who can understand part or almost all of it is increasing.

The survey results of left-behind children's demand for musical practice courses are shown in Figure 6.

Figure 6 shows that at the beginning of the experiment, most of the left-behind children's understanding of the music course is limited to singing and appreciation in the music class. After the four-month intervention, the left-behind children's cognition of the music class becomes sharper. The concept of performance and appreciation is added to music classes. This also just shows that musical practice classes can stimulate children's self-confidence and expression, making them more willing to show themselves.

### 3.4. Experimental Results Based on the Observation Method

Based on the observation of the number of bad behaviors of left-behind children in the musical practice classes, the statistical results are shown in Figure 7.

Figure 7 shows that after four months of experimental intervention, the frequency of left-behind children's bad behavior decreases significantly. As for the object competition, children's role in the musical is loved by everyone and recognized by teachers, and they know how to help and cooperate with each other. The number of physical conflicts with students drops to 0, indicating that the students begin to learn to control their behavior, and the number of other bad habits is also less and less.

### 3.5. Results of Mental Health Intervention of Musical Practice Classes

After four months of musical practice classroom intervention, the mental health of left-behind children is tested for the second time, and the test results are shown in Figure 8.

Figure 8 shows that after a period of intervention, the number of the left-behind children who choose the options of “frequently missing their parents, feeling lonely, having no confidence, lying, and feeling afraid, helpless and afraid” decreases, while the number of the left-behind children who choose the options of “frequently making more friends and being braver” increases significantly. The number of children who choose the options of feeling lonely, having no confidence, and telling lies decreases significantly. Thus, after four months of musical practice classroom intervention, the mental problems of left-behind children have been relieved significantly.

In short, musical practice classes can train children's oral expression ability, and cultivate them to help each other, cooperate, and bravely show their self-recognition. The help and cooperation in practical activities reduce loneliness and establish self-confidence. It plays a good role in the regulation and prevention of left-behind children's mental problems.

## 4. Conclusion

Health is the most important for children. Health not only means that there is no disease or disability in the body but also means a healthy mental state and social adaptability. A healthy child needs not only physical health but also mental health. Based on the questionnaire survey, the mental health states of left-behind children are studied, hoping to intervene in the mental problems of left-behind children through musical practice, which plays the role of prevention and regulation. Through the research, the following three conclusions are drawn: (1) Most left-behind children lack self-confidence and are timid and more likely to care about the remarks of others. (2) Left-behind children like music, singing, and music can bring them happiness, but many left-behind children are shy to perform and express themselves because of their introverted characters and timidity. (3) The practice class of musical drama can promote the left-behind children to help each other and cooperate in practice activities, reduce their loneliness, and establish their self-confidence.

Due to the limitations of research funding and other objective factors, this study only selected first- and second-year students as samples, and the sample was not comprehensive enough. The incomplete sample is the shortcoming of this study. In the future, the research field will be further broadened, and the intervention of psychological problems of left-behind children will be studied for other types of art forms.

## Figures and Tables

**Figure 1:** Companionship of left-behind children in the whole year (B shows the companionship by their parents, C shows the companionship by their grandparents, and D shows the companionship by others).

**Figure 2:** Mental health states of left-behind children.

**Figure 3:** Left-behind children's attitudes towards music classes.

**Figure 4:** Reasons why left-behind children like music lessons ((a) shows how left-behind children feel about music classes, (b) shows what left-behind children think they can learn from music lessons, and (c) shows what left-behind children like most about music classes).

**Figure 5:** Music knowledge of left-behind children.

**Figure 6:** Survey results of left-behind children's demand for musical practice course.

**Figure 7:** Statistical results of the observation method (B represents the total number of bad behaviors, C represents physical conflicts, D represents object competition, and E represents bullying).

**Figure 8:** Comparison of the effects of musical practice classroom intervention (BCD shows the mental states before the experiment, B1C1D1 shows the mental states after the experiment, B means often, C means sometimes, and D means not).

**Table 1:** Reliability statistics.

Cronbach's alpha	Cronbach's alpha based on normalized terms	Items
.804	.803	5

**Table 2:** KMO and Bartlett's test.

Sampling adequacy of Kaiser-Meyer-Olkin	Measure	0.657
Bartlett's sphericity test	Approximate chi-square	143.478
	Df	55
	Sig	.000

**Table 3:** Basic information of the left-behind children.

Gender	Number	Age (number)	Grandparent guardianship	Grandparents-in-law guardianship	Under the guardianship of others
Male	36	Less than 7 years old (29)	30	3	3
		7-8 years old (7)			
Female	22	Less than 7 years old (19)	19	2	1
		7-8 years old (7)			

## Data Availability

The data used to support the findings of this study are included within the article.
